# Maternal resveratrol consumption and its programming effects on metabolic health in offspring mechanisms and potential implications

**DOI:** 10.1042/BSR20171741

**Published:** 2018-03-09

**Authors:** Sheng Zheng, Qianyun Feng, Jing Cheng, Jia Zheng

**Affiliations:** 1 Tianjin University of Traditional Chinese Medicine, Tianjin, China; 2 Department of Pediatrics, The Second Teaching Hospital of Tianjin University of Traditional Chinese Medicine, Tianjin, China; 3 The Key Laboratory of Cardiovascular Remodeling and Function Research, Chinese Ministry of Education and Chinese Ministry of Health, The State and Shandong Province Joint Key Laboratory of Translational Cardiovascular Medicine, Shandong University Qilu Hospital, Shandong, China; 4 Department of Endocrinology, Peking University First Hospital, Beijing, China

**Keywords:** cardiometabolic health, offspring, pregnancy, Resveratrol consumption

## Abstract

A growing body of evidence has clearly demonstrated that maternal nutrition can strongly determine the susceptibility to the development of metabolic diseases in offspring. With the increasing prevalence of maternal overweight, obesity, and gestational diabetes mellitus, it yields enormous burden for individual and public health. Interventions during pregnancy have been proven to be challenging, with limited efficacy and low compliance. Resveratrol, as a natural polyphenolic compound, has a wide-range of beneficial properties, including potent antiobesogenic, antiatherosclerotic, and antidiabetic effects. However, the role of maternal resveratrol intake on metabolic health in offspring has not been extensively investigated. Therefore, the aim of this study was to review the effects of maternal resveratrol supplementation on metabolic health in offspring and its potential mechanisms.

## Introduction

The incidence of obesity and diabetes is increasing rapidly, placing a huge economic burden on society [1]. However, the pathogenesis of diabetes has not been fully illustrated. Emerging data show that perinatal nutrition consumption is a pivotal factor determining the susceptibility to metabolic disorders [2–4]. In particular, approximately one in six births is affected by gestational diabetes mellitus (GDM) reported by International Diabetes Federation Atlas in late 2017 [1]. The World Health Organization newly reported that 50% of women of childbearing ages, and 20–25% of pregnant women in Europe were affected by overweight or obesity [5]. As demonstrated by the “Developmental Origins of Health and Disease (DOHaD)” theory [6,7], obese mothers and women with GDM are associated with infant weight *z*-scores at birth and at 6 months [8], childhood obesity [9], and unhealthy body composition in adult offspring [10,11]. They are more likely to develop insulin resistance [12], type 2 diabetes [13,14] and even early childhood type 1 diabetes [15], and cardiovascular diseases [16] in adulthood.

## Interventions for metabolic health during pregnancy are limited

With the increasing prevalence of metabolic diseases during pregnancy, such as maternal obesity and GDM, it yields enormous burden for individual and public health [17]. Preventing obesity, insulin resistance, and type 2 diabetes during pregnancy has pronounced benefits [18]. Lifestyle interventions, including diet and exercise, have been widely used to prevent and treat abnormal metabolism during pregnancy [19]. However, it has proven to be challenging, with limited efficacy and low compliance. One meta-analysis indicated that diet and lifestyle interventions in pregnancy were able to reduce gestational weight gain; however, no effects on composite maternal and fetal outcomes were observed [20]. Poston et al. [21] showed that a behavioral intervention with diet and physical activity in obese mothers was insufficient to reduce the incidence of fetal macrosomia or to prevent GDM occurrence. Han et al. [22] showed that for women with GDM, there were no differences in adverse pregnancy outcomes among several kinds of dietary advice. Flynn et al. [23] showed that the methodological variability in dietary interventions to control gestational weight gain in pregnant women was large, which limited the ability to apply the evidence in clinical practice and develop clinical guidelines. Other management practices, such as medication therapy for GDM, are expensive and with side effects [24]. Therefore, alternative interventions for metabolic health during pregnancy are needed.

## Historical perspective of active compounds isolated from plants and herbs

Traditional Chinese Medicine (TCM), as an herbal medicine with a 2000-year-old history, has been widely used to treat diseases in most Asian countries [25]. The safety, efficacy, and mechanisms of most TCM have been clearly demonstrated, and compounds from dietary plants and herbs have been widely used in complementary and alternative medicine [26]. For example, artemisinin, as an important antimalarial drug, is mainly discovered and isolated from sweet wormwood [27]. In addition, approximately 50% of pharmaceutical drugs may be plant derivatives [28]. Salicylic acid, isolated from the willow tree, is the basis of the common drug, aspirin. Atropine, as a muscle relaxant, is isolated from nightshade plants, and morphine is extracted from the opium poppy [29]. In recent years, active compounds isolated from plants and herbs have been discovered, due to its multiple therapeutic capacities [25,30].

## Resveratrol and its roles in human health

Resveratrol, a polyphenolic compound (3,4′,5-trihydroxystilbene), is mostly isolated from grapes (Figure 1). It also naturally presents in a variety of plant foods such as peanuts and cranberries [31]. It indicates that resveratrol has a variety of beneficial health effects, such as anti-inflammatory [32], antioxidant [33], and anticarcinogenic [34] properties. Resveratrol also can ameliorate metabolic diseases [35], including cardioprotective, antiobesogenic [30], antiatherosclerotic [36], and antidiabetic [37] effects. A systematic analysis of 21 studies found that daily resveratrol consumption (≥300 mg/day) significantly reduced blood pressure, total cholesterol, and plasma glucose in obese subjects, with lower risks of cardiovascular diseases [38]. However, evidence about the effects of maternal resveratrol intake on metabolic health in offspring is limited. Therefore, we aimed to review the effects of maternal resveratrol consumption on metabolic health in offspring and its potential mechanisms underlying these programming effects.

**Figure 1:** The molecular structure of resveratrol isolated from grapes Resveratrol, a polyphenolic compound (3,4′,5-trihydroxystilbene), is mostly present in grapes. Resveratrol has a variety of beneficial health effects and exhibits several biological properties, including its cardioprotective, antiobesogenic, antiatherosclerotic, and antidiabetic effects.

## Maternal resveratrol consumption and metabolic health

### Evidence from clinical studies in human

The beneficial effects of resveratrol supplementation in humans are widely studied, but the studies about the effects of resveratrol intake during pregnancy on metabolic health in humans are limited. Several studies show that oral resveratrol is well absorbed and rapidly metabolized, without pronounced toxicity [39,40]. One clinical study was conducted to evaluate the metabolic effects of resveratrol in overweight pregnant women. It showed that resveratrol supplement (80 mg) reduced the incidence of GDM and improved the lipid profile and glucose blood level after 60 days [41]. It also showed that both the time and doses of blood pressure control were significantly reduced in preeclampsia patients who received resveratrol supplementation (50 mg each, up to five dosages) [42]. It suggested that maternal resveratrol intake has a beneficial effect in pregnant women. However, the evidence is limited and no information is available about the different effects of resveratrol depending on the dietary intake on pregnant women. Thus, more clinical studies with larger sample size are needed.

### Evidence from *in vivo* and *in vitro* experiments

#### Maternal resveratrol consumption and glucose metabolism

Animal experiments showed that maternal resveratrol consumption can improve glucose metabolism in pregnant females, as well as in offspring. Resveratrol supplementation throughout pregnancy was able to decrease maternal body weight, improve glucose tolerance, and increase blood flow volume in uterine artery, with lower triglyceride deposition in liver and decreased placental inflammation in nonhuman primates [43]. Using a genetic mouse model of GDM, it showed that resveratrol intake (10 mg/kg body weight per day) before pregnancy and during pregnancy significantly alleviated hyperglycemia, improved insulin resistance, increased fetal survival, and decreased body weight at birth. They further found that resveratrol enhanced adenosine monophosphate activated protein kinase (AMPK) activation and reduced glucose-6-phosphatase activity in pregnant C57BL/KsJ-Leptin (db/+) mouse, as well as the offspring [44]. Using human samples, Lappas et al. [45] investigated the effects of resveratrol incubation (50, 100, and 200 μmol/l) on insulin resistance and placental inflammation associated with GDM. It showed that resveratrol was able to ameliorate placental inflammation triggered by lipopolysaccharide (LPS), with decreased tumor necrosis factor (TNF), interleukin-6 (IL-6), and interleukin-8 (IL-8) gene expressions in human placentas. Recently, Tran et al. [46] found that treatment with resveratrol (200 μmol/l) significantly reduced the secretion and expression of proinflammatory cytokines, such as IL-6, interleukin-1α (IL-1α), interleukin-1β (IL-1β), IL-8, and monocyte chemoattractantprotein-1 (MCP-1) in human placenta and adipose tissue. It was able to restore the impaired insulin signaling and glucose uptake activity assessed by radio-labeled assay in skeletal muscles obtained from pregnant individuals. Thus, maternal resveratrol intake had a beneficial effect on glucose metabolism in pregnant females and offspring.

#### Maternal resveratrol consumption and its effects on lipid metabolism

Maternal resveratrol administration (0.2% diet) in pregnant mice increased energy expenditure and insulin sensitivity, which was associated with increased brown adipose activity and the browning of white adipose tissue [47]. Maternal resveratrol consumption (50 mg/l in the drinking water) during pregnancy and lactation reduced body weight, serum leptin level, visceral and subcutaneous adipose tissue weight, with females being more affected in offspring rats, indicating sexually dimorphic impact [48]. Franco et al. [49] also showed that maternal resveratrol intake (30 mg/kg body weight/day) decreased body weight and fat mass in offspring. It was able to reverse hyperleptinemia and improve hypothalamic leptin signaling. Resveratrol administration (100 mg/kg body weight) from embryonic day 3 to 12 prevented the occurrence of oxidative stress and apoptosis in embryos; it further decreased blood cholesterol level by 41.74% and triglyceride level by 60.64% in diabetic dams [50]. Thus, it indicated that maternal resveratrol intake was able to improve lipid metabolism in both dams and offspring.

#### Maternal resveratrol consumption and its effects on cardiovascular function

Maternal resveratrol supplementation (4 g/kg diet) during pregnancy and lactation alleviated the development of hypertension in adult offspring, with improved nitric oxide bioavailability in spontaneously hypertensive rats [51]. However, Moraloglu et al. [52] found that resveratrol intake (20 mg/kg per day) during the whole pregnancy did not decrease blood pressure, and did not result in a significant response in blood flows and placental pathology parameters in pregnant rats. Resveratrol consumption (4 g/kg diet) improved cardiac recovery from ischemia/reperfusion injury and attenuated superoxide levels in both male and female rat offspring exposed to prenatal hypoxia [53]. This variability in findings could be caused by variations in the different doses of resveratrol intake or the length of study duration. Thus, it suggests that the efficacy of distinct doses is needed to be evaluated and the best dosing should be determined in further studies. The relevant evidence of maternal resveratrol intake and metabolic health in both pregnant females and offspring are summarized in Table 1.

**Table 1:** Relevant studies about maternal resveratrol intake and metabolic health in offspring

Resveratrol consumption	Intervention period	Species	Beneficial effects on pregnant females	Beneficial effects on offspring	Potential mechanism	References
A Western-style diet supplemented with 0.37% resveratrol	Throughout pregnancy	Nonhuman primates	- Resulted in maternal weight loss and improved glucose tolerance	- Fetal pancreatic mass was enlarged by 42%	May be driven by an eNOS-dependent mechanism	Roberts et al. [43]
			- Increased uterine artery volume blood flow	- A 12-fold increase in proliferation		
			- Decreased placental inflammation and liver triglyceride deposition			
Oral gavage with resveratrol (10 mg/kg body weight per day)	Four weeks before pregnancy and during pregnancy	A genetic GDM model: C57BL/KsJ-Leptin (db/+) mouse	- Improved glucose metabolism, insulin tolerance, and reproductive outcome of the pregnant db/+ females	- Increased fetal survival and decreased body weight	- Enhanced AMPK activation	Yao et al. [44]
					- Reduced production and activity of G6Pase	
50, 100, and 200 μmol/l resveratrol incubation	6- and/or 24-h incubation	Human placenta	- Quenched inflammation induced by LPS	NA	- SIRT1 possessed anti-inflammatory actions	Lappas et al. [45]
200 μmol/l resveratrol incubation	20-h incubation	Human placenta, adipose tissue, and skeletal muscle	- Reduced the expression and secretion of pro-inflammatory cytokines IL-6, IL-1α, IL-1β, IL-8, and MCP-1 in human placenta and omental and subcutaneous adipose tissue	NA	- Restored the impaired insulin signaling pathway and insulin-mediated glucose uptake in human skeletal muscle	Tran et al. [46]
A high-fat diet with or without 0.2% (w/w) resveratrol	During pregnancy and lactation	C57BL/6 J mice	- Protected dams against body weight gain and fat accumulation	- Increased energy expenditure and insulin sensitivity	- Increased phosphorylated AMPKα levels, Sirt1, PRDM16, and other thermogenic genes protein contents	Zou et al. [47]
			- Reduced the concentrations of triglycerides and insulin	- Enhanced white adipose tissue browning		
Resveratrol (50 mg/l) in drinking water	During pregnancy and lactation	Wistar rats	- No difference in body weight at the end of lactation	- Reduced body weight, leptin, VAT and SCAT, with females being more affected	- Decreased fatty acid synthase expression in VAT	Ros et al. [48]
					- An antiadipogenic effect	
Resveratrol (30 mg/kg body weight/day)	8 weeks before mating and throughout gestation and lactation	Wistar rats	NA	- Decreased body weight, subcutaneous and visceral fat mass, and adiposity	- Increased p-STAT3 content in the hypothalamus	Franco et al. [49]
Resveratrol (100 mg/kg body weight) was administered by gavage feeding	10 days (from day E3 to E12)	Sprague Dawley rats	- Decreased lipid accumulation including cholesterol by 41.74% and triglyceride by 60.64% and increased HDL in diabetic dams	- Prevented both oxidative stress and apoptosis in embryos	- Stimulation of the extrinsic and intrinsic pathway	Singh et al. [50]
					- May attenuate the expression of HMG-CoA reductase	
Resveratrol-supplemented diet (4 g/kg diet)	From gestational day 0.5 until postnatal day 21	Spontaneously hypertensive rat	- Had no effect on blood flow patterns in the maternal uterine arteries	- Mitigated the development of hypertension in adult offspring	- Improved nitric oxide bioavailability	Care et al. [51]
20 mg/kg per day and twice daily	During the whole pregnancy	Wistar albino rats	- Did not decrease blood pressure	NA	NA	Moraloglu et al. [52]
			- No changes in blood flows and placental pathology parameters			
Resveratrol supplementation (4 g/kg diet)	For 9 weeks following weaning	Sprague–Dawley rats	NA	- Improved cardiac recovery from ischemia/reperfusion injury	- Unclear, without AMPK–ACC signaling activation	Shah et al. [53]
				- Attenuated superoxide levels		

Abbreviations: ACC, acetyl-CoA carboxylase; AMPK, adenosine monophosphate activated protein kinase; E, embryonic; eNOS, endothelial nitric oxide synthase; G6Pase, glucose-6-phosphatase; GDM:, gestational diabetes mellitus; HDL, high-density lipoprotein; HMG-CoA, hydroxy-3-methyl-glutaryl (HMG)-CoA reductase; IL-1α, interleukin-1α; IL-1β, interleukin-1β; IL-6, interleukin-6; IL-8, interleukin-8; LPS, lipopolysaccharide; MCP-1, monocyte chemoattractantprotein-1; NA, not available; PRDM16, PR domain containing 16; p-STAT3, phosphorylated-signal transducer and activator of transcription 3; SCAT, subcutaneous adipose tissue; SIRT, sirtuin; VAT, visceral adipose tissue.

#### Possible harmful effects of resveratrol

In addition to the above beneficial effects of resveratrol, detrimental effects of resveratrol should also be considered. Studies that reported possible harmful effects of resveratrol are limited. Roebrts et al. [43] found that, in stark contrast with the other seemingly beneficial effects to the placenta and developing fetus, a dramatic increase in fetal pancreatic mass and exocrine proliferation, independent of an increase in islet mass, following maternal resveratrol supplementation in nonhuman primates which is clinically concerning. Klink et al. [54] showed that resveratrol was associated with significantly worse survival with LAPC-4 (the human CaP cell line) tumors and caution should be advised in using resveratrol for patients. Further studies about other possible harmful effects of resveratrol should be conducted.

### Potential mechanisms of maternal resveratrol consumption and metabolic health in offspring

Taken together, the above studies suggest that maternal resveratrol intake protects against hyperglycemia, insulin resistance, dyslipidemia, and cardiac function in pregnant females, as well as their offspring. However, the molecular mechanisms are not clearly elaborated. It is speculated that “developmental programming” may be the underlying mechanism that can elucidate maternal nutrition and metabolic health in offspring [55]. Several potential points can explain the beneficial effects of maternal resveratrol consumption on offspring, which are summarized in Figure 2. First, resveratrol can decrease inflammation reaction in placental and normalize embryonic oxidative stress level [43], due to its anti-inflammatory [32], antioxidant [33] properties. Second, it can reverse hyperleptinemia and improve hypothalamic leptin signaling in offspring [49]. Another possible mechanism is epigenetic modification [56]. Our previous studies showed that epigenetics can link early life nutrition and cardiometabolic health in later life [57–60]. It demonstrated that resveratrol was able to modulate histone H3 on lysine 9 (H3K9) methylation and acetylation in the zygotic pronuclei [61]. Gestational resveratrol exposure induced breast cancer-1 (BRCA-1) promoter hypermethylation and reduced BRCA-1 expression in mammary tissue of rat offspring [62]. However, whether the role of maternal resveratrol consumption on the offspring is due to adaptive responses to improved glucose and lipid metabolism in mothers, or is the direct result of resveratrol transfer through the placenta or the mother’s milk is still unclear. There have been no reports, however, on whether resveratrol crosses the placental barrier. One study showed that as a polyphenol, administration of resveratrol has vasodilator effect on isolated human umbilical vein *in vitro* [63]. Jang et al. [64] showed that resveratrol is beneficial against diabetes-induced embryonic malformation, we therefore might cautiously assume that it does cross the placental barrier. Thus, further studies focusing on this point and the molecular mechanisms in depth are warranted.

**Figure 2:** Maternal resveratrol consumption and its beneficial effects on metabolic health in offspring It is speculated that “Developmental Programming” is the underlying mechanism because it can link maternal nutrition and metabolic health in offspring. Several potential points could explain the beneficial effects of maternal resveratrol consumption on offspring. First, resveratrol can decrease inflammation reaction in placental and normalized embryonic oxidative stress level, due to its anti-inflammatory and antioxidant properties. Second, it was able to improve hypothalamic leptin signaling in offspring with central nervous system regulation. Another possible mechanism is epigenetic modification, including methylation and acetylation, thus regulate gene expressions.

## Conclusions

In summary, pregnancy period is the critical time window of offspring/embryo growth and development. Perinatal nutrition consumption can determine the susceptibility of developing metabolic diseases in adulthood. Interventions during pregnancy are challenging, with limited efficacy and low compliance. Our review suggests that maternal resveratrol consumption during pregnancy has beneficial effects on metabolic health in both pregnant females and offspring. More importantly, the safe and easy implementation of resveratrol consumption has been widely accepted. A broad understanding of the role of resveratrol supplementation during pregnancy can provide critical hints for the early prevention and treatment of metabolic diseases during pregnancy, and thus ensure a healthier future for the mothers and offspring.

## Abbreviations

AMPK: adenosine monophosphate activated protein kinase
BRCA-1: breast cancer-1
GDM: gestational diabetes mellitus
IL: interleukin
LPS: lipopolysaccharide
MCP-1: monocyte chemoattractantprotein-1
TCM: Traditional Chinese Medicine
TNF: tumor necrosis factor
